The article "Innovation of Ideological and Political Education Management of College Students Based on IOT Big Data Technology in a Wireless Network Environment" was retracted in 2023. Reasons: unreliable results or conclusions; lack of ethics approval or compliance; concerns about the data; concerns about the peer review.

# Innovation of Ideological and Political Education Management of College Students Based on IOT Big Data Technology in a Wireless Network Environment

**DOI:** 10.1155/2022/9585760

**Published:** 2022-06-09

**Authors:** Zheng Du

**Affiliations:** Jinhua Education College, Jinhua, 321000 Zhejiang, China

## Abstract

Universities are not only the front line of national ideological and political works but also the gathering place of national talent training, which is of far-reaching significance to the national strategic development, and it is vital to do a good job of ideological and political education in universities for the construction and development of the country. “The university has become a place where wireless network technology can be used. The paper examines the current state of mobile learning in the United States and abroad, explains the principles for developing a mobile ideological and political learning system, designs and studies the system's overall structure and functional modules, and shows how the system's application can replace traditional ideological and political learning methods, allowing students to improve their ideological and political abilities using mobile devices.

## 1. Introduction

With the rapid development of information technology and the information industry, the demands on network communications are increasing and wireless networking technology is making up for the shortcomings of traditional network technology and a radio can be used to great effect both over long distances and in close proximity [1]. The uses are very similar to those of limited networks. The major difference lies in the transmission medium [2]. The use of radio technology instead of a network can be used as a backup to a wired network. Ideological and political education is to analyze the different kinds of human needs and then distinguish between reasonable and unreasonable needs and different levels of needs, so as to carry out ideological and political education and solve the problem of unmet needs or the problem of different needs being met one after another [3]. The leading role of the ideological and political education of university students is to play a positive role in promoting the comprehensive, coordinated, and sustainable development of students [4–7].

The Internet has gradually replaced the radio and television as the main channels for people, especially young people, to obtain information in their daily lives [8]. People have recognized the convenience of the Internet, and the ease of access to wireless networks implies that university students have more flexibility of choice [9]. Wireless network technology provides university students with access to information not only in terms of time and space but also in terms of content and form, providing them with a rich and complex range of sources from mobile phones, tablets, laptops, and desktop computers. While network technology is developing at a rapid pace, the network environment is not optimistic, especially as many unscrupulous elements are promoting extremist ideas on the network or taking advantage of students' gullible personalities to commit network fraud [10].

It is more likely to be incited by socially undesirable ideas. Wireless network technology has not only brought the people the convenience of updating their thoughts [11]. Many unscrupulous elements precisely use college students' ears to think simple and other characteristics, propagating their bad speech to achieve its profiteering to disturb the social order [12–15].

The teaching mode is more conservative compared to other disciplines. The content is more serious. There is a lot of theoretical content. Students find it difficult to understand. The efficiency of the classroom is low, and many of the ideological and political theory classes have become “disaster areas” where students are absent from the class. Students are active and have a strong sense of thinking. With the development of the times, students receive a huge amount of information, although they are young [16]. They are young, but their minds are mixed with a variety of ideas. To carry out ideological and political education work in colleges and universities means to do the work in the field of ideas and to guide students to receive advanced theoretical knowledge of the Communist Party of China. It is not a matter of forceful indoctrination, which would only cause resentment among students [17–20].

The paper arrangements are as follows:

Section 2 describes the ideological and political education in the environment of IoT.  Section 3 defines the ideological and political education system design and implementation.  Section 4 examines the intelligent recommendation algorithms for student development models based on learning trajectories.  Section 5 analyzes the experimental results.  Section 6 concludes the paper.

## 2. Ideological and Political Education in the Environment of IoT

This section discusses the analysis of the current situation and defines the research significance.

### 2.1. Analysis of the Current Situation

Since the 1970s, the emphasis on intelligent teaching systems has increased. In particular, Western countries such as the USA have attached particular importance to the development of intelligent education systems [21]. These countries have strong economic power, and science and technology have driven the development of intelligent market industries, as well as optimizing the design of intelligent education systems. With the advancement of the Internet of things technology, intelligent teaching systems are gradually being applied to school teaching in the United States, primarily for physics, chemistry, and other science services [22]. Intelligent science services can be simulated through the system to improve professional teaching services, and with the advancement of the Internet of things technology, intelligent teaching systems are gradually being applied to school teaching, with great success. Compared with this, China's intelligent teaching system still needs a breakthrough to further strengthen and improve the service function of the intelligent teaching system to provide effective services for actual teaching. At present, China's intelligent teaching system has made a breakthrough in technology, mainly in artificial intelligence technology to assist teachers in their daily work [23]. Combined with traditional education, intelligent education is a new type of education system based on computer technology, which emphasizes the organic combination of intelligent technology and education, teachers and teaching, etc. It can improve the education system, thus strengthening the quality of teaching and improving students' interest in learning and enabling systematic evaluation, allowing students to learn independently and understand and master students' abilities, especially in ideological and political education, which must be pushed forward to strengthen students' ideological and political competencies [24, 25].

### 2.2. Research Significance

It is true that our country already has numerous online ideological and political education websites. But there are still many problems that have been revealed, which seriously affect the use of the system by students. First of all, there are regional differences. The selectivity of the teaching textbooks in the intelligent system leads to different textbooks and learning contents, and different regions use different versions of teaching materials and training programs, leading to educational ideas and regions being in “opposition.”

## 3. Ideological and Political Education System Design and Implementation

### 3.1. Overall System Design

The ideological and political education system, according to the requirement analysis, is typically employed as a learning aid and must ensure that the user experience is effective while also ensuring that its objectives are performed to the greatest extent possible. In order to simplify the overall design requirements and to research on the existing system structure, the author starts from the role of the ideological and political education system crowd; it can be concluded that there are three types of users in the system, namely, system administrators, teacher users, and student users. Each of them has a different function. By integrating the functions that have overlapping needs, the following modules are finally obtained, which are described in detail in Figure 1.

### 3.2. Function Implementation

#### 3.2.1. Student Management

Student management is more targeted and based mainly on the student learning content. Ideological and political education needs to take into account students' ability to listen, read, and write. It should enable registration and login and the viewing and modification of personal information. Also, as the core content, students can view courseware, video tutorials, test questions, and complete online quizzes. They can also view website announcements and post online responses to messages, etc. These functions certify that students can access the learning end of the system to learn effectively and achieve the resolution of independent learning, as shown in Figure 2.

In the module ideological and political education system for students to learn the main module, students first have to register and select the appropriate class and subclass learning; students can be combined with the actual ideological and political levels of communication with the class teacher, at the same time, they can be based on the stage. The system may generate reports based on student grades, and students and teachers can efficiently analyze deficiencies and provide comments on study hours based on detailed data. In addition, students can upload teaching materials outside of the platform system to increase the extracurricular learning content, giving full play to the function of the ideological and political education system and thus improving students' ideological and political performance. The message board can post online, reply to messages, etc. Students can ask questions, communicate with teachers, and appear as a learning forum, while students can learn about grades, class assignments, news announcements, etc. on the message board, enabling them to keep abreast of their learning, consult with classmates and teachers, exchange learning experiences, and make full use of the system's functions [26, 27].

#### 3.2.2. Teacher Management/Administrator Management

Teachers and administrators can act as the “decision makers” for the background functions. Both teachers and administrators have the ability to add, delete, and enter. The administrator can manage teacher information, student information, course information, data information, etc. in the system, as shown in Figure 3.

The administration centre is used by teachers to manage users, manage courseware, add assignments, and manage online questions and other basic information management, and the administration message board has functions such as forum management and replying to messages. Therefore, the login functions of teachers and administrators have similarities and differences. Teachers mainly manage learning tests, teaching aids, and teaching resources, while administrators mainly add, modify, and delete information [28, 29].

## 4. Intelligent Recommendation Algorithms for Student Development Models Based on Learning Trajectories

### 4.1. Data Collection and Mining

According to the results of the intelligent advice and the preferences of the students, the school completes the redesign of the student learning course system, provides for the appropriate professional learning, and realizes the innovation of the student training mode. The data source for this recommendation system is student information, book information, and borrowing information, and the differentiation and humanization of students' practical ties are enhanced through the use of intelligent analytic technology.

### 4.2. Selection of Recommendation Algorithms

The interest-based recommendation algorithm uses item-based collaborative filtering (item CF for short). The core of the algorithm is to use user behavior data to calculate the similarity between items and to make personalized recommendations based on the user's historical behavior and the item similarity matrix. When predicting user interests, it is important to consider weighing the user's recent behavior more heavily and adding temporal validity information to the user recommendation results. The core of the recommendation algorithm based on the learning trajectory is to mine the background data from students' history of book borrowing and Internet browsing on the campus for a more personalized and specialized course system, making student training more targeted and improving the quality of student training.

The item CF algorithm consists of two main steps.

- Calculate the similarity between items [30]

(1) $$\begin{array}{c} W\left(ij\right)=\frac{\left|N\left(i\right)\cap N\left(j\right)\right|}{\sqrt{\left|N\left(i\right)\right|\left|N\left(j\right)\right|}},\\ P\left(u,j\right)=\underset{i\in S\left(j,k\right)\cap N\left(u\right)}{\sum }W\left(j,i\right)*r\left(u,i\right). \end{array}$$

### 4.3. Improvements to Item CF

#### 4.3.1. Consider the Popularity of the Item [31]

In the calculation of item similarity, active users contribute more to the item similarity than inactive users and it can also be considered that the more popular the item is, the more it contributes to the calculation of item similarity. The formula for calculating item similarity is as follows:

(2) $$\begin{array}{c} w\left(i,j\right)=\frac{\sum_{u\in N\left(i\right)\cap N\left(j\right)}\left(1/\log\left(1+\left|N\left(u\right)\right|\right)\right)}{\sqrt{\left|N\left(i\right)\right|\left|N\left(j\right)\right|}}, \end{array}$$

where |*N* (*u*)| denotes the number of items of interest to user *u*.

#### 4.3.2. Time Context-Dependent Item CF Algorithm

When calculating item similarity, it is also important to consider the effect of temporality. The closer to the current time, the more similar the item is to the user, and the formula for calculating similarity is as follows:

(3) $$\begin{array}{c} w\left(i,j\right)=\frac{\sum_{u\in N\left(i\right)\cap N\left(j\right)}\left(1/\log\left(1+\alpha *\left|T_{u_{i}}-\right|T_{u_{j}}\right)\right)}{\sqrt{\left|N\left(i\right)\right|\left|N\left(j\right)\right|}}. \end{array}$$

The recent behavior is more indicative of the user's current interest than the previous behavior, where the user's interest in the item *P* (*u*, *i*) is calculated using the following equation:

(4) $$\begin{array}{c} P\left(u,i\right)=\underset{j\in S\left(i,k\right)\cap N\left(u\right)}{\sum }W\left(i,j\right)*r\left(u,j\right)*\frac{1}{1+\alpha \left(T_{0}-T_{u_{j}}\right)}. \end{array}$$

## 5. Experimental Results

In the experiment, taking the software engineering course system as an example, the abovementioned recommendation algorithm is applied to improve and update the course system, which can obtain a course system more in line with individual characteristics.

As illustrated in Figure 4, the recommendation of online education is still hampered by transmission rate limitations, the use of teaching courseware, network speed issues, and other factors that impede learners' ability to learn online. As a result, in the Internet of things technology environment, an integrated examination of the ideological and political education system design is also required, so the paper uses based on B/S system framework structure construction and 3-layer logic structure, to further improve the security and applicability of the system, B/S system framework structure through the Java language programming run, can make it in the browser side, the server side of a large number of computing processing, easy to develop and maintain. Formation of the browser-side (B) - release instructions - server-side (S) - calculation results - The 3-layer structure under the B/S system can form a highly cohesive and low-coupling state, further improving the performance of the ideological and political education system.

As seen in Figure 5, we believe that learning is tedious and ineffective. The “double-edged sword” of wireless network technology can be efficiently used by ideological and political education in higher education to construct an online learning platform, for example, by opening a WeChat account. Through the WeChat subscription number, we can publish weekly or monthly summaries of social and current affairs and the key arrangements of ideological and political work; we can also build a web space, upload the main contents of ideological and political education in the form of a journal, and require students to study online.

Figure 6 depicts the distribution of students' learning interests as a useful tool for sorting out Internet information sources. Ideological and political educators in colleges and universities should pay greater attention to network information media and stay up to date on diverse topics in order to guide college students in determining what is right and incorrect. Many network information publishers are unconcerned about information's accuracy and scientificity. As a college ideological and political educator, you should pay more attention to the information. In the classroom or during the evening roll call, they should analyze and explain inaccurate or radical comments to help students judge right and wrong. For example, during a certain period of time, students should not be misled by bad information on the Internet. For example, during a certain period of time, the international relations between China and Japan were tense. Many students on university campuses have been incited by “anti-Japanese” sentiments on the Internet. They were encouraged to take part in illegal demonstrations and even to vandalize Japanese cars and electrical shops. Ideological and political educators in universities should make use of evening roll calls and class meetings to analyze the situation. Guide students to be rational and patriotic. Avoid a situation that gets out of hand.

For example, they can check more classes, communicate more with college teachers, and strictly discipline the use of mobile phones in class, as shown in Figure 7, so as to reduce the chances of students using their hand percussion in class and restore good classroom order. The majority of ideological and political educators in higher education are student ideological and political counsellors, who have the most contact with students and can make use of opportunities such as evening roll calls or class meetings to strengthen education and propaganda for students to fully understand the autonomy and conscientiousness of learning.

## 6. Conclusions

With the development of Internet of things technology, education tends to be more technological and informational development, the application of the network education platform for ideological and political teaching has been achieved, and there is no doubt that the intelligent development of education is a change to the traditional ideological and political teaching mode. The system not only provides students with individualized instruction, such as online learning, online testing, downloading, online question answering, and other services, but also serves as a showcase for wireless network technology as a gathering place for young talent. The work of ideological and political education in colleges and universities should make good use of this “double-edged sword,” so that it can play a positive role in promoting ideological and educational works.

## Figures and Tables

**Figure 1:** Overall design of the ideological and political education system.

**Figure 2:** Diagram of student management.

**Figure 3:** Diagram of teacher management/administrator management functions.

**Figure 4:** Diagram of the recommendation algorithm.

**Figure 5:** Student learning outcomes in Civics.

**Figure 6:** Distribution of learning interests.

**Figure 7:** Student-teacher fit.

## Data Availability

The datasets used during the current study are available from the corresponding author upon reasonable request.
